# Potential Mechanisms of Shu Gan Jie Yu Capsule in the Treatment of Mild to Moderate Depression Based on Systemic Pharmacology and Current Evidence

**DOI:** 10.1155/2022/3321099

**Published:** 2022-08-22

**Authors:** Taiping Li, Tian Qiu, Yanyan Zeng, Bing Kang, Xianglong Tang, Ning Yang, Hong Xiao

**Affiliations:** ^1^Department of Neuro-Psychiatric Institute, The Affiliated Nanjing Brain Hospital of Nanjing Medical University, Nanjing 210029, China; ^2^Department of Pharmacy, The Affiliated Nanjing Brain Hospital of Nanjing Medical University, Nanjing 210029, China; ^3^Department of Pharmacy, Quanzhou Maternity and Children's Hospital, Quanzhou 362019, China; ^4^Department of Traditional Chinese Medicine, The Affiliated Nanjing Brain Hospital of Nanjing Medical University, Nanjing 210029, China

## Abstract

**Background:**

Shu Gan Jie Yu (SGJY) capsule has a good effect on relieving depressive symptoms in China. However, the mechanism of action is still unclear. Therefore, systemic pharmacology and molecular docking approaches were used to clarify its corresponding antidepressant mechanisms.

**Methods:**

Traditional Chinese Medicine Database and Analysis Platform (TCMSP), the Encyclopedia of Traditional Chinese Medicine (ETCM), and Swiss Target Prediction servers were used to screen and predict the bioactive components of the *SGJY* capsule and their antidepressive targets. Mild to moderate depression (MMD) related genes were obtained from GeneCards and DisGeNET databases. A network of bioactive components-therapeutic targets of the *SGJY* capsule was established by STRING 11.5 and Cytoscape 3.9.0 software. Gene function and Kyoto Encyclopedia of Genes and Genomes (KEGG) pathway enrichment analyses were performed by utilizing Database for Annotation, Visualization, and Integrated Discovery (DAVID) platform. Active components were taken to dock with the hypothetical proteins by iGEMDOCK and SwissDock, and the docking details were visually displayed by UCSF Chimera software. Then, the related research literature of the *SGJY* capsule was reviewed, summarized, sorted, and analyzed, including experimental evidence and clinical experience.

**Results:**

Seven active components and 45 intersection targets were included in the study. PPI network had genuinely uncovered the potential therapeutic targets, such as *AKT1, HSP90AA1, ESR1, EGFR,* and *PTGS2*. KEGG pathway analysis showed that the mechanism of the *SGJY* capsule on MMD was mainly involved in the PI3K-Akt signaling pathway.

**Conclusions:**

In this study, we have successfully predicted the biochemically active constituents, potential therapeutic targets, and comprehensively predicted the related drug-gene interaction of the *SGJY* capsule for treating MMD and provided a basis for subsequent experiments.

## 1. Introduction

Depression is one of the most disabling disorders worldwide with poor quality of life. It affects human social function, and imposes a heavy economic burden on individuals, families, communities, and countries. Due to the increasing social pressure and the role of various other factors, mild to moderate depression (MMD), as an early stage of depression, shows a trend of younger age [1]. Currently, selective serotonin reuptake inhibitors (SSRIs) have been widely used in clinical treatment, but their therapeutic effectiveness is only limited at ∼65% [2]. Thus, more effective drugs with less adverse reactions are expected to be developed in the future. Nowadays, traditional natural herbs are usually used to relieve depression and balance emotions [3].

Systematic review and meta-analysis have provided effective evidence that Shu Gan Jie Yu (*SGJY*) capsule showed an effective intervention for essential hypertension patients with insomnia, anxiety or depression in recent years. And it is widely used in the treatment of MMD. The *SGJY* capsule mainly concludes two Chinese herbs, *Acanthopanax senticosus* (Rupr. & Maxim.) Harms (ASH) and *Hypericum perforatum* L. (HPL). The antidepressant mechanism of ASH may be mediated *via* the central monoaminergic neurotransmitter system and cAMP response element-binding (CREB) protein expression. Therefore, administration of ASH may be beneficial for patients with depressive disorders [4]. HPL, widely known as *St. John's wort*, is commonly used in clinical practice for its antidepressant properties, as well as anxiolytic its properties[5]. In addition, HPL extract is effective in treating MMD and is safer than SSRIs [6]. Although the *SGJY* capsule has achieved good clinical efficacy in the treatment of MMD, its mechanism of action is still unclear.

With the rapid development of chemoinformatics and bioinformatics, systematic pharmacology, a technology based on computer simulation, has become a developing interdisciplinary. It applies network pharmacology to indicate the molecular mechanisms of Traditional Chinese Medicine (TCM), and has been widely used in screening bioactive components in TCM. In general, systemic pharmacology technology could evaluate the pharmacological effects and reveal the underlying relationship among active components, potential targets, and multiple diseases [7].

In this study, a systemic pharmacology-based strategy combined with molecular docking approach had been employed to predict bioactive components, potential gene targets, and related signal pathways of the *SGJY* capsule on depression treatment. The flowchart of research approach is shown in Figure 1.

## 2. Methods

### 2.1. Screening for Active Components of the *SGJY* Capsule

Traditional Chinese Medicine Database and Analysis Platform (TCMSP, https://www.tcmsp-e.com/) and the Encyclopedia of Traditional Chinese Medicine (ETCM, https://www.tcmip.cn/ETCM/index.php/Home/) were used to screen components of ASH and HPL [8]. The screening criteria were set as oral bioavailability (OB) greater than or equal to 30% and drug-likeness property (DL) greater than or equal to 0.18 [9]. The molecular structure was reconfirmed by PubChem platform (https://pubchem.ncbi.nlm.nih.gov/) and saved in .mol2 and SMILES format for further study.

### 2.2. Potential Targets Prediction

Active components were submitted to Swiss Target Prediction platform (https://www.swisstargetprediction.ch/) based on SMILES format with parameter Probability ≥0.6 in prediction results in order to obtain high-quality targets [10]. “*Homo sapiens*” was used as selected species. After removing duplicate genes, potential targets related with active components of the *SGJY* capsule were obtained. MMD-related targets were collected individually from the DisGeNET (https://www.disgenet.org/home/) and GeneCards (https://www.genecards.org/) databases with the keywords “psychotic depression, mental depression, depressive disorder, mild depression, and moderate depression.” All the targets were standardized in the UniProt database (https://www.uniprot.org/).

### 2.3. Network Construction and Gene Analysis

*SGJY*-related and MMD-related targets were all imported into the Venny 2.1 system (https://bioinfogp.cnb.csic.es/tools/venny/). The intersection targets were selected as the potential targets for further analysis. A protein–protein interaction (PPI) network was constructed by using the STRING 11.5 platform (https://string-db.org/), “Organism” was set to “*Homo sapiens*.” An interaction with medium confidence (0.4) was collected. The network was visually displayed by the Cytoscape 3.9.0 software. Then GO function and KEGG enrichment analyses were performed with the DAVID platform (https://david.ncifcrf.gov/tools.jsp). The identifier and species were selected as “*official_gene_symbol*” and “*Homo Sapiens*,” respectively. The enrichment results, including molecular functional (MF), cell component (CC), biological process (BP), and KEGG pathway enrichment, were obtained and visualized by using imageGP platform (https://www.ehbio.com/ImageGP/index.php/Home/Index/index.html) as the bubble graph with *p* value <0.05 [11].

### 2.4. Molecular Docking

Crystal structures of core proteins were obtained from the RCSB Protein Data Bank (PDB, https://www.rcsb.org/) with high resolution and score. Water molecules were removed from the structure. Potential candidate components of the *SGJY* capsule in .mol2 format were taken as ligands. Molecular docking was mainly completed by iGEMDOCK 2.1 with default parameters. Afterward, the most potential protein with associated active ingredients at the low energy was used to dock on the SwissDock platform (https://www.swissdock.ch/docking/), and the results were visually displayed by the UCSF Chimera 1.15 software.

### 2.5. Literature Collection and Analysis

Literature search was performed *via* PubMed database (https://pubmed.ncbi.nlm.nih.gov/) with the term “Shu gan jie yu.” All relevant literature were collected, organized, categorized, and divided into experimental evidence and clinical practice.

## 3. Results

### 3.1. Collection and Screening Bioactive Components of the *SGJY* Capsule

Ten active components of the *SGJY* capsule were screened out *via* the TCMSP and ETCM database with the thresholds of OB ≥ 30% and DL ≥ 0.18 properties (Table 1), while ASH and HPL have a common compound named 3-epi-beta-sitosterol (PubChem CID 12303645). However, 3-epi-beta-sitosterol, ethyl oleate, and acanthoside B were excluded because of no gene interaction in the network. Finally, 7 bioactive molecules were collected for further analysis, including betulinic acid, sesamin, kaempferol, cianidanol, luteolin, (+)-epicatechin, and quercetin.

### 3.2. Determination of Common Targets

After excluded duplicate data, 116 candidate targets of main components were collected, 7041 and 1747 MMD-related targets were identified from GeneCards and DisGeNET databases, respectively. 45 intersection targets were shown as a Venn diagram (Figure 2).

### 3.3. PPI Network Construction and Analysis

Forty-five intersection genes correlated with MMD were analyzed by the STRING database, and PPI network was established (Figure 3(a)). A total of 45 nodes and 70 edges were embodied with the average node degree 8.53 and *p* value <0.01. The most-connected targets were *AKT1, HSP90AA1, ESR1, EGFR, PTGS2, GSK3B, MMP9, MMP2, IGF1R, KDR, APP, MCL1, PIK3R1,* and *MAPT* with larger degree (degree > 10), as shown in Table 2 and Figure 3(b). The network of herbs-components-targets was constructed, including 2 herbs, 7 components, and 45 potential targets, in which the blue hexagons correspond to the putative targets and bioactive components are in pink (Figure 4).

### 3.4. Gene Function and KEGG Pathway Enrichment Analyses

To further capture the relationships between the terms, the DAVID platform was used to perform gene function and KEGG pathway analyses with *p* value <0.05. The main biological processes contained signal transduction, negative regulation of apoptotic process, and protein autophosphorylation (Figure 5(a)). Cellular components mainly involved plasma membrane, cytoplasm, and nucleus (Figure 5(b)). Protein, ATP, and identical protein binding were the main molecular functions of intersection genes (Figure 5(c)). The mechanisms of the *SGJY* capsule in the treatment of MMD included PI3K-Akt, Ras, and estrogen signaling pathways (Figure 5(d)). Among them, the PI3K-Akt pathway was the most potential signaling pathway.

### 3.5. Molecular Docking

PPI network construction and gene analysis indicated that the potential targets of the *SGJY* capsule against MMD were based on their degree. They were selected to dock with 7 active components (betulinic, cianidanol, (+)-epicatechin, kaempferol, luteolin, quercetin, and sesamin). Fluoxetine, which was a SSRI and widely used in clinical practice, was used as a positive control [12]. The lowest binding energy shows the most stable combination. The value of fitness was used to evaluate the binding level. The total energy was regarded as a predicted pose in the binding site, which included Van Der Waal (VDW), hydrogen bonding (H-bond) and electrostatic energy, so *E*_total_ = *E*_VDW_ + *E*_H-bond_ + *E*_electrostatic_. It was interesting to note that most compounds had a better bonding ability to potential targets than fluoxetine, as shown in Figure 6. Moreover, (+)-epicatechin, kaempferol, luteolin, quercetin, and sesamin were all closely bound to protein *MMP9*, and sesamin had the better bonding mode with the *MMP9* protein than fluoxetine based on binding energy (Figure 7).

### 3.6. Literature Collection and Analysis

#### 3.6.1. Experimental Evidence of the *SGJY* Capsule

Shu Gan Jie Yu capsule mainly contains two Chinese herbs, *Acanthopanax senticosus* (Rupr. & Maxim.) Harms (ASH) and *Hypericum perforatum* L. (HPL). Many evidences show that ASH and HPL play an important role in the treatment of MMD.

Jin et al. found that ASH extract significantly elevated the levels of 5-hydroxytrylamine, norepinephrine, and dopamine in the whole brain of mice and up-regulated the level of CREB protein. It might exert antidepressant effects *via* the central monoaminergic neurotransmitter system and CREB protein expression [13]. *In vitro* studies had shown that ASH extract significantly increased the cell viability, suppressed the apoptosis of PC12 cells, and up-regulated CREB protein expression. Neuroprotective effect might be one of the acting mechanisms that accounts for the *in vivo* antidepressant activity of ASH [14]. The induction of HO-1 expression protected cells against glutamate-induced neuronal cell death. ASH extract could regulate HO-1 expression through the p38-CREB pathway and translocation of Nrf2, and played an important role in the generation of antineuroinflammatory and neuroprotective responses [4]. Moreover, it had beneficial effects on depression behaviors and restored both altered c-fos expression and hypothalamic-pituitary-adrenal (HPA) activity which associated with stress, and may be a novel agent for the treatment of stress-related disorders [15].

HPL, popularly called *St. John's wort*, is used as a medicinal plant for MMD, and is more effective than placebo or some antidepressant drugs. Di Pierro, et al. found that multifractionated hypericum extract has better clinical outcomes in subjects with depression without determining an increased risk of toxicity or reduced tolerability [16]. HPL could regulate the genes that control HPA axis function and influence, like conventional antidepressants. Thus, at least in part, it plays stress-induced effects on neuroplasticity and neurogenesis [17]. For patients with mild to moderate depression, *St John's wort* has comparable efficacy and safety when compared to SSRIs [18]. Most of HPL extracts have been shown to be significantly more effective than placebo with at least similar efficacy and better tolerability compared to standard antidepressant drugs. It is a safe and effective way to treat MMD over long periods of time with less adverse effects, and seems especially suitable for a relapse prevention [19–21].

#### 3.6.2. Clinical Practice of the *SGJY* Capsule

The *SGJY* capsule is widely used in clinical practice and has achieved very good clinical results in MMD. Clinical efficacy and safety of the *SGJY* capsule in patients with acute myocardial infarction and depression. Significantly lower adverse event rate was observed in the Shu Gan Jie Yu group. The *SGJY* capsule has a reliable effect and high safety in patients with depression [22]. In addition, it is very effective for treatment of senile depression [23].

The *SGJY* capsule is also an effective intervention for essential hypertension patients with insomnia, anxiety, and depression [3]. Yao et al. found that the *SGJY* capsule significantly reduced the depressive symptoms and improved cognitive functions in poststroke depressive patients through alteration of brain dynamics [24].

## 4. Discussion

Seven bioactive components of the *SGJY* capsule, including betulinic, cianidanol, (+)-epicatechin, kaempferol, luteolin, quercetin, and sesamin, had been successfully obtained by systemic pharmacology strategy. Recent studies also confirmed the antidepressant effects of these compounds. Kaempferol and quercetin had been reported to relieve symptoms of depression and exhibited antidepression effects through acting on *interleukin-6* (IL6), mitogen-activated protein kinase 1 (MAPK1), signal transducer, and activator of transcription 3 (STAT3) and transcription factor AP-1 (JUN) [25]. Betulinic produced a significant antidepressant-like effect [26]. Cianidanol, also called (+)-catechin, together with kaempferol and quercetin showed potential capacity in depression management [27]. Luteolin could prevent both neuroimmune responses and behavioral abnormalities including major depressive disorder, which was induced by visceral inflammation [28]. Sesamin inhibited chronic unpredictable mild stress (CUMS)-induced mice depressant-like behaviors and anxiety, which retained immobility and prevented stress-induced decrease of 5-HT and NE in the striatum and serum. Moreover, sesamin treatment significantly prevented CUMS-induced neuroinflammation by inhibiting over-activation of microglia and expressions of inflammatory mediators including *iNOS, COX-2, TNF-α,* and *IL-1β* in stressed mice hippocampus and cortex [29]. Therefore, multiple active components of the *SGJY* capsule may exert therapeutic effects on MMD.

PPI network analysis showed that 14 core targets correlated bioactive components had been determined, such as *AKT1, HSP90AA1, ESR1, EGFR, PTGS2, GSK3B, MMP9, MMP2, IGF1R, KDR, APP, MCL1, PIK3R1,* and *MAPT*. Some studies had reported that the *AKT1* gene was strongly associated with antidepressant treatment [30, 31], which further confirmed our results. And *PTGS2* [32, 33], *EGFR* [34], *ESR1* [35, 36], *APP* [37], *IGF1R* [38, 39], *KDR* [40], *GSK3B* [41, 42], *MAPT* [43], and *PIK3R1* [44] played very important roles in prevalence and progression of depression. It was verified that *HSP90AA1* was up-regulated in patients with depression, which correlated with elevated levels of *VEGF, VEGFR2, PI3K,* and *AKT1* [45]. Some studies showed that *MMP-2* and *MMP-9* genes had relative lower expression on both mRNA and protein levels in depression [46, 47]. *MMP9*, a key protein for extracellular matrix degradation, was significantly correlated with depressive symptoms [38, 39]. Our study found that most of the bioactive components of the *SGJY* capsule had good binding capacity to *MMP9*, which indicated that *MMP9* played a very important role on *SGJY*-treated MMD.

Signal transduction has been reported to be closely involved in antidepressant treatment. Gene function and KEGG results indicated that the main molecular mechanism of the *SGJY* capsule in the treatment of MMD was the PI3K-Akt signaling pathway, *KDR, CDK6, IGF1R, EGFR, INSR, GSK3B, HSP90AA1, PIK3CG, MCL1, PIK3R1*, and *AKT1* genes were enriched in it. Quercetin, luteolin, and kaempferol had been confirmed to be effective in the treatment of MMD by *in vivo* experiments. The potential PI3K-Akt signaling pathway, a classic signaling pathway in cells, closely relates to the biological process of depression [43, 48]. It regulates fundamental cellular functions such as transcription, translation, proliferation, growth, and survival. In addition, the *SGJY* capsule might exert therapeutic effects on MMD *via Ras*, estrogen, and *Rap1* signaling pathways. Homologous Ras-family small GTPases, including *Ras, Rap2,* and *Rap1*, played a different role and presented signal diversity and specificity. Ras signals long-term potentiation *via* endoplasmic reticulum *PI3K* and lipid raft *ERK*, whereas *Rap2* and *Rap1* signal depotentiation and long-term depression *via* bulk membrane *JNK* and lysosome *p38MAPK*, respectively [49]. Thus, Ras-family small GTPases related signaling pathways, including *Ras-Raf-MAPK* [50], *Ras-ERK-MAPK* [51], and *Rap1-MKK3/6-p38 MAPK* [52], may be involved in explaining the disease etiology, the clinical symptom, and treatment response of stress-induced depression [53]. Increasing evidence had been manifested that the disturbances of estrogen signaling pathway occurred in psychiatric disorders, especially in female depression [54]. Hence, the role of multiple signaling pathways is under consideration. Further study is warranted to reveal the relationship between core targets activated by potential bioactive components of the *SGJY* capsule and different related signaling pathways.

Due to the limitations of compounds screening and accuracy of target prediction, the results obtained in this study are general [55]. Although there is some evidence, many *in vivo* and *in vitro* experiments are still needed for verification. In short, our study portrayed the ground view of the *SGJY* capsule in the treatment of mild to moderate depression.

## 5. Conclusion

In this study, seven bioactive components of the *SGJY* capsule have been identified by a systemic pharmacology-based strategy and the intersection targets corresponding to these components and their therapeutic mechanism of MMD have been revealed in detail by the PPI network and pathway enrichment analyses. The result of molecular docking showed that sesamin had a better bonding mode with the *MMP9* protein than fluoxetine. In general, bioactive components and the main therapeutic mechanism of the *SGJY* capsule in the treatment of MMD were successfully predicted, which might provide valuable guidance for further pharmacological research of the *SGJY* capsule on MMD.

## Figures and Tables

**Figure 1:** The research flowchart of antidepressant mechanism of the *SGJY* capsule.

**Figure 2:** Diagram of overlapping target genes between the *SGJY* capsule and MMD.

**Figure 3:** PPI network analysis. (a) PPI network of targets constructed using STRING 11.5. Nodes represent proteins. Edges represent PPIs. (b) The network constructed by Cytoscape 3.9.0 according to the enrichment degree; the more lines, the more connections.

**Figure 4:** The network of herbs-components-targets. The red shows the Chinese herbs of the *SGJY* capsule, the cyan displays the active components of the *SGJY* capsule, and the blue shows the most potential targets of the *SGJY* capsule in the treatment of MMD. Furthermore, the density of lines represents the interaction relationship between different protein targets.

**Figure 5:** GO enrichment and KEGG pathway analyses. (a) Biological process (BP) terms, (b) cellular component (CC) terms, and (c) molecular function (MF) terms of GO enrichment analysis (top 10). (d) KEGG pathway enrichment (top 10). The color of the dot is displayed in a gradient from red to green according to the ascending order of the *p* value, while the size is arranged according to the ascending order of the number of gene counts. The longitudinal axis represents the name of different terms or pathways, and the transverse axis shows the percentage of the number of enriched genes to the total number of genes. *p* value <0.05.

**Figure 6:** Molecular docking results. Red color represents low docking score, and blue represents high docking score. The lowest value indicates the most stable conformation (kcal/mol).

**Figure 7:** The best binding modes of sesamin (a) and fluoxetine (b) with *MMP9* protein by SwissDock. Visualization is performed using UCSF Chimera.

**Table 1:** Basic information of the main active components of the *SGJY* capsule.

Herbs	PubChem CID	Chemical name	OB (%)	DL
ASH	12303645	3-Epi-beta-sitosterol	36.91	0.75
	5363269	Ethyl oleate	32.40	0.19
	64971	Betulinic acid	55.38	0.78
	72307	Sesamin	56.55	0.83
	443024	Acanthoside B	43.35	0.77

HPL	12303645	3-Epi-beta-sitosterol	36.91	0.75
	5280863	Kaempferol	41.88	0.24
	9064	Cianidanol	54.83	0.24
	5280445	Luteolin	36.16	0.25
	182232	(+)-Epicatechin	48.96	0.24
	5280343	Quercetin	46.43	0.28

**Table 2:** Potential targets of the *SGJY* capsule against MMD (degree > 10).

No.	UniProt ID	Gene names	Protein names	PDB ID	Degree
1	P31749	AKT1	RAC-alpha serine/threonine-protein kinase	7NH5	28
2	P07900	HSP90AA1	Heat shock protein HSP 90-alpha	3O0I	24
3	P03372	ESR1	Estrogen receptor	5FQV	23
4	P00533	EGFR	Epidermal growth factor receptor	5GNK	22
5	P35354	PTGS2	Prostaglandin G/H synthase 2	5F19	20
6	P49841	GSK3B	Glycogen synthase kinase-3 beta	6Y9S	18
7	P14780	MMP9	Matrix metalloproteinase-9	6ESM	17
8	P08253	MMP2	72 kDa type IV collagenase	3AYU	15
9	P08069	IGF1R	Insulin-like growth factor 1 receptor	1P4O	15
10	P35968	KDR	Vascular endothelial growth factor receptor 2	6GQQ	13
11	P05067	APP	Amyloid-beta precursor protein	4PWQ	13
12	Q07820	MCL1	Induced myeloid leukemia cell differentiation protein Mcl-1	6OQD	13
13	P27986	PIK3R1	Phosphatidylinositol 3-kinase regulatory subunit alpha	2IUG	13
14	P10636	MAPT	Microtubule-associated protein tau	6ODG	11

## Data Availability

The data used to support the findings of this study are available from the corresponding author upon request.

## Abbreviations

ASH: *Acanthopanax senticosus* (Rupr. & Maxim.) Harms
BP: Biological process
CC: Cell component
CREB: CAMP response element-binding
CUMS: Chronic unpredictable mild stress
DAVID: Database for annotation, visualization, and integrated discovery
DL: Drug-likeness
ETCM: Encyclopedia of Traditional Chinese Medicine
GO: Gene Ontology
HB: Hydrogen bond
HPA: Hypothalamic-pituitary-adrenal
HPL: *Hypericum perforatum* L.
HT: 5-hydroxytryptamine
KEGG: Kyoto encyclopedia of genes and genomes
MF: Molecular function
MMD: Mild to moderate depression
MMP-2: Matrix metalloproteinase 2
MMP-9: Matrix metalloproteinase-9
NE: Norepinephrine
OB: Oral bioavailability
PDB: Protein data bank
PI3K-Akt: Phosphatidylinositol 3-kinase-protein kinase B
PPI: Protein-protein interaction
ROS: Reactive oxygen species
SDF: Structure-data file
SGJY capsule: Shu Gan Jie Yu capsule
SSRIs: Selective serotonin reuptake inhibitors
TCM: Traditional Chinese medicine
TCMSP: Traditional Chinese medicine database and analysis platform.
